# Influence of Implant Surface Topography on Primary Stability in a Standardized Osteoporosis Rabbit Model Study

**DOI:** 10.3390/jfb6010143

**Published:** 2015-03-18

**Authors:** Hiroshi Oue, Kazuya Doi, Yoshifumi Oki, Yusuke Makihara, Takayasu Kubo, Vittoria Perrotti, Adriano Piattelli, Yasumasa Akagawa, Kazuhiro Tsuga

**Affiliations:** 1 Department of Advanced Prosthodontics, Graduate School of Biomedical and Health Sciences, Hiroshima University, 1-2-3 Kasumi, Minami-ku, Hiroshima 734-8553, Japan; E-Mails: hiroshi-o@hiroshima-u.ac.jp (H.O.); yos-oki14@hiroshima-u.ac.jp (Y.O.); yusuke0318@hiroshima-u.ac.jp (Y.M.); kubocky@hiroshima-u.ac.jp (T.K.); tsuga@hiroshima-u.ac.jp (K.T.); 2 Department of Medical, Oral and Biotechnological Sciences, Chieti-Pescara University, Chieti-Via dei Vestini, 31, Chieti 66100, Italy; E-Mails: v.perrotti@unich.it (V.P.); apiattelli@unich.it (A.P.); 3 Department of Prosthetic Dentistry School of Dentistry, Ohu University, 31-1 sankakudo, Kooriyama, Fukushima 963-8611, Japan; E-Mail: akagawa@den.ohu-u.ac.jp

**Keywords:** primary stability, osteoporosis, glucocorticoid, implant surface, rabbit model

## Abstract

Evaluating primary stability is important to predict the prognosis of dental implant treatment. Primary stability is decreased in a low bone density site such as osteoporosis. However, it is difficult to apply in small animal and the effect of the different implant surface topography for the primary stability at low bone density site has not yet fully been investigated. The purpose of the present study was to evaluate the influence of implant surface topography on primary stability in a standardized osteoporosis animal model. Six rabbits underwent ovariectomy and administrated glucocorticoid to induce an osteoporosis model. Sham-operations were performed in additional six rabbits. Implants with machined or oxidized-surfaces were inserted into the femur epiphyses and insertion torque (IT) and implant stability quotient (ISQ) were measured. In sham model, the IT and ISQ did not differ significantly between the both implant. However, the IT value of oxidized-surface implant was significantly higher than that of the machined implant in the osteoporosis model. Meanwhile, ISQ did not significantly differ between the machined and oxidized-surfaced implants. In conclusion, the IT of implants is higher with rough than with smooth surfaces but that there are no differences in ISQ value between different surfaces in a standardized osteoporosis bone reduced rabbit model.

## 1. Introduction

Dental implant therapy has been successfully used to replace missing teeth, particularly in healthy bone [1,2]. The long-term success of implant therapy depends on the achievement of favorable primary stability at implant placement. Primary stability is influenced by various factors, and the two main factors affecting primary stability are density and quantity of bone at the implant site and implant design [3,4]. 

It is well known that primary stability in low bone density sites is decreased. Recently, the problems faced with osteoporosis have received attention in not only the orthopaedic field but also dental implant therapy. Osteoporosis is a skeletal disease that causes systematic loss of bone density and strength [5]. Therefore, low bone density caused by osteoporosis might lead to decreased primary stability. Indeed, osteoporosis may be a risk factor for implant failure [6]. 

The screw-type implant aids easy acquisition of primary stability and is now standard. Moreover, implant surface topography is a key factor in the achievement of osseointegration. The most common modification of implant topography is surface roughness; this is achieved by acid etching, sandblasting, or oxidization. Anodic oxidization modifies the chemical composition and the degree of crystallinity [7]. Oxidized titanium implants, such as the TiUnite™ produced by spark anodized, have a moderately rough implant surface that enhances the speed of osseointegration by stimulating bone growth, thereby reducing the risk of implant failure during the early healing phase [8]. 

The development of low bone density animal models has been essential in studies of bone mass as well as the development of new drugs for osteoporosis [9]. Ovariectomy is recognized as the gold standard in experimental animal osteoporosis models using rats or mice. However, insertion of commercialized dental implants is difficult in these models because the bone quantity is insufficient for implant placement. Although rabbit model have been used to evaluate osseointegration or implant stability of commercialized dental implants [10], rabbits are remarkably resistant to conventional strategies for inducing bone loss, and thus ovariectomy is seldom successful. For this reason, the influence of surface topography on primary stability at low bone density sites remains unverified *in vivo*. Recently, an experimental osteoporosis model using rabbits has been established in which significant bone loss is achieved within a short period by combining ovariectomy with glucocorticoid administration [11]. Glucocorticoids mainly affect bone quality by decreasing bone formation through osteoblastogenesis reduction and increased osteoblast and osteocyte apoptosis. The analysis of various surface modification or novel biomaterials with commercialized dental implant has been performed in healthy animals [12]. In the future, the significance of these analyses in osteoporotic animal will be demanded in research fields of implant material and biomaterial. This experimental rabbit osteoporosis models enable investigation of dental implants inserted in a standardized low bone density site. 

The purpose of this study was to evaluate the influence of surface topography on primary stability in an osteoporosis rabbit model.

## 2. Results and Discussion

### 2.1. Results

#### 2.1.1. Insertion Torque

The insertion torque (IT) value was higher in the sham than osteoporotic (OP) models in both the rough-surfaced and smooth-surfaced groups. In the sham model, IT of the rough group was 33.1 ± 6.1 N·cm and that of the smooth group was 26.1 ± 5.7 N·cm, with no significant difference between 2 groups. In the OP model, the IT value of the rough group was 13.6 ± 3.6 N·cm and that of the smooth group was 7.1 ± 2.7 N·cm. A significant difference was found between the rough-surfaced and smooth-surfaced groups (*P* < 0.05) (Figure 1). 

**Figure 1:** (**a**) Insertion torque (IT) value of Sham model group was higher than that of the osteoporotic (OP) model group (*P* < 0.05); (**b**) In the OP model, IT value of rough group was higher than that of smooth group (*P* < 0.05); (**c**) In the sham model, there was no significant difference between the groups.

#### 2.1.2. Resonance Frequency Analysis

The implant stability quotient (ISQ) was higher in the sham than OP model in both the rough and smooth groups. In the sham model, the ISQ values of the rough and smooth implants were 73.4 ± 3.1 and 70.3 ± 8.6, respectively. The corresponding values in the OP model were 63.6 ± 4.5 and 56.3 ± 14.4, respectively. In both models, no significant difference was observed between rough and smooth implants (Figure 2).

**Figure 2:** (**a**) Implant stability quotient (ISQ) value of the Sham model group was higher than that of the OP model group (*P* < 0.05); (**b**,**c**) In both models, ISQ values were no significantly different between the smooth and rough groups.

#### 2.1.3. Mechanical Strength of Bone

The maximum mechanical bone strength of the sham model (295.9 ± 32.9 N) was significantly higher than that of the OP model (202.7 ± 25.5 N, *P* < 0.05) (Figure 3). 

**Figure 3:** The bars represent maximum loads in the sham model and OP model, and the error bars indicate the corresponding standard deviations (SDs). The maximum load of the sham model (295.5 ± 32.9 N) was significantly higher than that of the OP model (202.7 ± 25.5 N) (*P < 0.05).

### 2.2. Discussion

The IT and ISQ values of the Sham model were higher than that of the OP model. The IT value was higher with rough surface topography than smooth surface topography in the osteoporosis model, meanwhile, the ISQ value did not differ significantly between these two groups. 

Implant stability is regarded as indication of the mechanical connection between the implant surface and surrounding bone [13]. Superior primary stability at implant placement leads to long-term success of implant treatment and indication of immediate loading [4,8]. The acquisition of primary stability depends on the bone quality and quantity [14], as well as the implant surface topography and design. At sites with poor bone density, such as in osteoporosis, the primary stability is decreased. 

Although rabbits have been widely used in studies involving dental implants, ovariectomy alone might be insufficient to induce osteoporosis in an osteoporosis rabbit model [11,15]. An experimental rabbit model of osteoporosis combining the effects of ovariectomy and glucocorticoid administration has been reported to show significant bone loss within a short period. This osteoporosis model is consistent, easy to be induced, and highly reproducible [15]. The decline in oestrogen levels induced by ovariectomy increases osteoclast recruitment, differentiation, and survival; consequently, bone resorption exceeds bone formation. Furthermore, glucocorticoid induces decreased bone formation through osteoblastogenesis reduction and increased osteoblast and osteocyte apoptosis [16]. Increased osteoclastic resorption and decreased new bone formation in cortical and trabecular bones, due to glucocorticoid administration and oestrogenic deprivation, have been previously demonstrated in the experimental osteoporosis rabbit model used in this study [15]. With dual-energy X-ray analysis, bone mineral density was significantly decreased in an ovariectomy model with glucocorticoid administration compared with a normal model. In addition, according to the results of mechanical strength analysis in the present study, the maximum mechanical bone strength of the OP model was lower than that of the sham model. Therefore, the OP model demonstrated a loss of bone density and mechanical strength. Commercialized dental implant cannot be applied in the mouse or rat models. However, this experimental rabbit osteoporosis model could be used for the investigation of the various surface modification or biomaterials with commercialized dental implants in the future study. 

Implant stability is considered an important indicator of the success of an implant [14,17]. Intraoperative methods for assessment of primary stability drilling resistance, insertion torque force, and resonance frequency analysis (RFA). Measurement of IT is useful for these the resistance force between implant thread and cortical bone site and is a reflection of the entire bone condition at the placement site. During implant insertion, IT is calculated as the torsional loading between bone interface and implant thread. A high IT is associated with superior primary stability and could reduce micro-motion after placement. IT value is generally affected by cortical bone thickness of the placement site [18]. The study results revealed that IT was higher in the sham than OP model in both the rough-surface and smooth-surface groups. IT values did not differ significantly between both groups in the sham model. On the other hand, IT of the rough group was significantly higher than that of the smooth group in the OP model. This finding suggests that the resistance of torsional load induced during implant placement is greater with a rough-surface thread than smooth-surface thread at sites with reduced bone density and thickness of cortical bone due to glucocorticoid administration. Therefore, implant surface topography could affect IT in the OP model but not in the sham model. It is considered that both groups could gain high friction during implant insertion in the sham model because bone density and thickness was sufficient for implant placement. Therefore, if bone quality at the implant placement site is appropriate, IT is affected by placement site condition rather than implant surface topography. Taken together, results of present study suggest that bone density and quantity are important factors for primary stability and rough-surface topography is predictably effective with low bone density at the implant placement site.

The ISQ of successfully stabilized implant is reported to range from 57 to 82 [19]. In this present study, ISQ values of the sham model were recorded as >60, indicating that implants in both groups were adequately stabilized at the placement site. ISQ values of the OP model were significantly lower than those of the sham model. There were no significant differences in the ISQ values between the rough-surface and smooth-surface groups in the sham model, whereas the ISQ values in the rough group tended to be higher than those in the smooth group in the OP model. This may mean that the ISQ value reflects the bone attachment area between the implant thread surface and corresponded surrounding bone. 

Compared with machined implants, oxidized titanium implants, such as the TiUnite™ implant, have been shown to have superior stability because bone healing or formation is accelerated after implant placement. Oxidized modified surface modification is beneficial for predictable achievement of osseointegration; however, it has been reported that ISQ values at implant placement are not significantly different between oxidized and machined surfaces [8]. In the present study, ISQ values immediately after implant placement did not differ significantly between rough and smooth groups in both the sham and OP models, it indicates that implant surface topography did not affect RFA measurements significantly. RFA might be mainly affected by bone quality and quantity around the implant and might be unable to detect differences in implant surface topography. Further, ISQ measurements alone might not be useful as a method to evaluate primary stability in certain placement site bone conditions such as decreased trabecular bone. Favorable ISQ and IT measurements do not necessarily indicate perfect primary stability. In addition, the relationship between ISQ and IT is not clear [18,20,21]. Accordingly, it is highly recommended that multiple methods should be used to assess primary stability in clinical situations. The influence of implant surface topography on primary stability in standardized bone-reduced site has not been fully investigated so far. Therefore, the results of this study could provide beneficial knowledge as to measurement of primary stability on osteoporosis. 

## 3. Experimental Section 

### 3.1. Ethics

This study was approved by the Research Facilities Committee for Laboratory Animal Science, Hiroshima University School of Medicine, Hiroshima (#A01-10).

### 3.2. Study Design and Animals

The study design of the animal procedure is shown in Figure 4. Twelve female New Zealand White rabbits (age, 17 weeks; body weight, 3.0–3.5 kg) were used in this study. Glucocorticoid-induced OP model animals were prepared according to previously described methods [11]. Animals were randomly selected for ovariectomy or sham operation (*n* = 6 in each model). Two weeks after ovariectomy, the six animals received intramuscular injections of glucocorticoid (methylprednisolone acetate, 1 mg/kg/day; Depo-Medrol^®^, Pfizer, Tokyo, Japan) for 4 consecutive weeks. The six sham-operated rabbits did not receive glucocorticoid and represented the non-induced osteoporotic model (sham model).

**Figure 4:** Design of the animal experiment.

Twelve oxidized surface-modified titanium dental implants (Brånemark system, MkIII TiUnite™, 3.75 mm diameter, 7 mm length, Nobel Biocare, Gothenburg, Sweden; Figure 5a) and 12 machined-surface titanium dental implants (Brånemark system, MkIII, 3.75 mm diameter, 7 mm length, Nobel Biocare, Gothenburg, Sweden; Figure 5b) were used in this study. The average surface roughness of the machined surface implant (smooth group) is 0.9 µm and of the oxidized surface (rough group) is 1.1 µm [22]. 

**Figure 5:** SEM image of the surface topography at the implant thread portion. (**a**) The surface of the oxidized implant; (**b**) The surface of the machined implant.

### 3.3. Measurement of Primary Stability

All procedures were performed under anesthesia with sodium pentobarbital (10 mg/kg, i.v.; Somnopentyl, Kyoritsu Seiyaku Corporation, Tokyo, Japan). 

All implant sockets were prepared according to the Brånemark protocol in the manufacturer’s instructions in the distal epiphysis of the knee joint of both femurs. Briefly, after the knee joint was exposed, a surgical micro-motor (Osseocare 2000^®^, Nobel Biocare, Gothenburg, Sweden) with rotary speed not exceeding 800 rpm was used for consecutive application of a 2.0 mm round drill, 2.0 mm twist drill, 3.0 mm pilot drill, 3.0 mm twist drill, and countersink drill. After implant socket preparation, the implant was inserted until the color indicator was level with the bone ridge. The maximum IT during the insertion was recorded by digital torque gauge (BTG-E100CN, Tonichi, Tokyo, Japan). After implant insertion, resonance frequency analysis (RFA) was performed using an Osstell^®^ (Osstell AB, Gothenburg, Sweden) to measure the ISQ (Figure 6). Measurements were done 3 times from 2 different directions, and the values obtained for each implant were averaged. The ISQ measurements were carried out according to previous study [23].

**Figure 6:** The measurement of implant stability quotient was performed using an Osstell^®^. The measurement was performed 3 times along both short and long axes to obtain average values in the placed implant.

### 3.4. Analysis of Mechanical Strength of Bone

Three-point bending tests were carried out according to previous study [24]. After the animals had been sacrificed, tibias of the OP and sham models were harvested and samples of bone 60.0 mm long were prepared by cutting 25.0 mm and 85.0 mm from the proximal end. A load was applied to the sample until the sample fractured (cross-head speed, 1 mm/min). Then, maximum load was recorded as the mechanical strength of the bone.

### 3.5. Statistical Analysis

Data of IT, ISQ and maximum load are presented as mean ± standard deviation (SD). Statistical analysis of the data was performed using Student’s *t*-test. Statistically significant differences were accepted as *P* < 0.05.

## 4. Conclusions 

In conclusion, the present study indicates that in a standardized bone reduced animal model, IT values of rough-surface implants are higher than those of smooth surface implants, and that there are no differences in ISQ measurements between different surfaces. Further studies in osteoporosis models might be expected to be conducted both *in vitro* and *in vivo,* including in the clinical situations. The osteoporosis rabbit model with ovariectomy and glucocorticoid administration appears beneficial for further experimental study of commercialized dental implants in osteoporosis. 
